# Surface modification of TiO_2_ nanoparticles with biodegradable nanocellolose and synthesis of novel polyimide/cellulose/TiO_2_ membrane

This article has been retracted.

**DOI:** 10.1016/j.jcis.2016.11.043

**Published:** 2017-04-01

**Authors:** Hashem Ahmadizadegan

**Affiliations:** Department of Chemistry, Isfahan University of Technology, Isfahan, Iran

**Keywords:** Polyimide, Cellulose, TiO_2_, Bionanocomposite, Gas permeation

## Abstract

In this paper, novel polyimide/cellulose/TiO_2_ bionanocomposites (PI/BNCs) were prepared via a simple and inexpensive ultrasonic irradiation process. PI was synthesized by direct polycondensation reaction of novel monomer dianhydride with 4-(2-(4-aminophenyl)-1,1,1,3,3,3-hexafluoropropan-2-yl)benzenamine. Due to the high surface energy and tendency for agglomeration the surface of nanoparticles was modified with cellulose. PI/BNCs containing 5, 10, and 15% of cellulose/TiO_2_ (BNCs) were successfully fabricated through ultrasonic irradiation technique. The obtained PI/BNCs were characterized by Fourier transform-infrared (FT-IR) spectroscopy, thermogravimetry analysis, X-ray powder diffraction, field emission-scanning electron microscopy (FE-SEM), and transmission electron microscopy (TEM). Thermogravimetric analysis data indicated an increase thermal stability of the PI/BNC polymers in compared to the pure polymer. From TEM image of PI/BNCs it can be found that the surface modified TiO_2_ with diametric size of less than 50 nm, uniformly dispersed in the obtained PI matrix. The results obtained from gas permeation experiments with a constant pressure setup indicated that adding cellulose/TiO_2_ to the polymeric membrane structure increased the permeability of the membranes.

## 1 Introduction

Bionanocomposites as a promising class of hybrid materials are derived from natural and synthetic polymers and organic–inorganic fillers at the nanoscale [1], [2], [3]. These materials are impacting on diverse areas, in specific, biomedical applications [4]. The essential question that has fascinated biomedical researchers from the beginning has thus been how to design and control material properties to achieve a specific biological reply [5], [6]. Scientists have usually sought help from chemistry in answering this question through synthesis of novel polymers based materials or the choice of reactives. In this mode, the biocompatibility of cellulosic compounds has been extensively studied due to the wide application as polymer in biomedical devices [7], [8], [9]. Cellulose nanofiber possess high surface to volume ratios, which means that they have a highly reactive and readily functionalizable surface [10], [11].

Polymeric nanocomposite membranes for gas separation represent a recognized technology for hydrogen recovery, nitrogen generation and carbon dioxide separation or capture from raw natural gas, since they provide an excellent properties processability balance and environmentally friendly path to achieve these processes [12], [13], [14], [15], [16], [17]. The gas separation behaviour of a membrane is described by the Robeson selectivity-permeability upper-bound relationship which has been regarded as an empirical criterion. However, the trade-off between gas permeability and selectivity exists as an objective for the study of membranes [18]. Many efforts have been done to enhance the permeability and selectivity of polymeric membranes [19], [20], [21], [22], [23], [24], [25], [26]. One method is to fabricate mixed matrix membranes or nanocomposite (NC) membranes. The NC membranes composed of incorporated nanoparticle (NP) fillers into a polymer matrix are of promising strategies for overcoming the limit of the Robeson upper bound [27], [28], [29], [30], [31], [32]. They could combine the outstanding properties of incorporated NPs and processability of the base polymers. To the best of our knowledge, there have been few studies that utilized metal oxides in membrane based gas separation applications. Between various metal oxides, TiO_2_ NPs are one of the multifunctional inorganic semiconductors with excellent optical, catalytic and electronic properties. This turns them into potentially attractive materials for production of TiO_2_-polymer NC membranes.

Aromatic polyimides are considered as one of the most significant modules of high performance polymers with a wide variety of applications from engineering plastics in aerospace industries to membranes in gas separation due to their exceptional mechanical strength and thermal stability, good electrical and optical properties as well as chemical resistance to many solvents [33], [34]. PIs bearing trifluoromethyl group (–CF_3_) substituent have drawn much attention because of significant enhancements in the polymer properties. Actually, the existence of a bulky —CF_3_ group in the polyimide structure has been shown to impart steric congestion which leads to producing soluble PIs with more free volume [35].

In order to reduce the environmental pollution caused by polymers, attempts are being made to modify their structures by blending or combining them with other biodegradable materials [36], [37]. Hence, the combination of polymers with cellulosic materials as, for example, blends, composites, nanocomposites and so on, are important areas of current research. There are very few reports of PI/cellulose/TiO_2_ nanocomposite formation by polymerization technique. The production of BNCs has gained increasing attention in recent years. Cellulose, one of the world’s most abundant, natural and renewable biopolymer resources, is widely present in various forms of bio-mass, such as plants. In cellulosic plant fibers, cellulose is present in an amorphous form, but is associated with crystalline phases through both intermolecular and intramolecular hydrogen bondings in which cellulose does not melt before thermal degradation [38]. Cellulose is organized in fibrils, which are aligned parallel to each other, surrounded by a matrix of lignin and hemicellulose. The properties of cellulose including mechanical state, low density and biodegradability [39] depend on the type of cellulose which is present. Owing to the abundance of hydroxyl groups existent on the surface of cellulose nanocrystals, reactive BNCs can be modified with different chemical groups to accomplish the expected surface modification like esterification and silylation or polymer grafting, which could successfully functionalize BNCs and facilitate its dispersion into different polymer matrices [40]. Therefore, BNCs is considered as one of the ideal nano-reinforcing agents for polymer matrices (including water soluble and water-insoluble polymer systems) and has been used into many polymer matrices to produce reinforced nanocomposites [41]. In addition, low density, low energy consumption, inherent renewability, biodegradability and bio-compatibility are also good advantages of environmentally-friendly BNCs [42]. Because of good dispersion of BNCs in water [43], fabrication and application of hydrogels including NCC without modification have many advantages versus other nanofillers such as polymer and metal nanoparticles. The improved interface between nanofillers and polymer matrix is beneficial to the properties of polymer-based nanocomposites. In nanocomposites, hydrogen bonding between BNCs and polymer matrix plays an important role in determining polymer-BNCs interaction [44].

There are different processing methods, sol–gel, microwave assisted method, ultrasonic irradiation and molecular capping, have been employed to form finely dispersed TiO_2_ nanoparticles in either organic or inorganic matrix. Ultrasonic irradiation is a moderately new but quite well established method which has been commonly used in preparing nanocomposites. Ultrasonic wave scattered modified nanostructure TiO_2_ particles in the polymer matrix. Compared to the conventional microwave method, the ultrasound method has attracted a great attention because it sharply reduces the overall processing time, increases the product yield and improves the quality of the product [45], [46], [47].

In this present investigation, in order to obtain solution-processable PI and PI/BNCs bionanohybrid films with higher T_g_ and enhanced gas separation properties, we therefore designed and synthesized a novel PI and PI/BNC membranes derived from new dianhydride monomer. In order to prevent agglomeration of nanoparticles and improve the dispersion of nanoparticles the TiO_2_ nanoparticles were treated with Cellulose nanofiber to introduce organic functional groups on the surface of TiO_2_. Then novel PI and PI/BNCs were synthesized under ultrasonic irradiation conditions. The resulting novel PI/BNCs are characterized by several techniques.

## 2 Experimental

### 2.1 Equipments

Carbon, hydrogen and nitrogen content of the compounds were determined by pyrolysis method by Vario EL (Elementar, Germany) elemental analyzer. FTIR spectra of the monomers and polymers were recorded from a NEXUS 870 FTIR (Thermo Nicolet) spectrophotometer at room temperature and humid free atmosphere using KBr pellets. ^1^HNMR spectra were recorded on a Bruker 500 instrument (Switzerland) using DMSO-*d*_6_ solvents. Inherent viscosities (η_inh_) of this PI in DMAc solvent were measured at about 0.5 g/dL concentration with an Ubbelohde viscometer at 31 ± 0.5 °C. Gel permeation chromatography (GPC) was performed with a Waters instrument (Waters 2414) and tetrahydrofuran (THF) was used as an eluent (flow rate 0.5 mL min^−1^). Polystyrene was used as a standard and a RI detector was used to record the signal in GPC. Glass transition temperatures (T_g_) were read at the middle of the transition in the heat capacity from the second heating scan. Thermogravimetric analysis (TGA) of the polymer sample was measured on a Netzsch TG 209F1 instrument at a heating rate of 10 °C min^−1^ innitrogen and air atmosphere. Differential scanning calorimetric (DSC) analysis was performed on a PE Diamond DSC instrument at a heating rate of 10 °C min^−1^ in nitrogen atmosphere. X-ray diffractometer (Philips Xpert MPD, Germany) with Cu Ka radiation (λ = 1.540 Å) was employed to determine the structure of newly synthesized polymers. Bragg angles ranged from 10 to 80° at the speed of 0.051 min^−1^. The operating current and voltage were maintained at 30 mA and 40 kV, respectively. The mechanical properties were measured on a Testometric Universal Testing Machine M 350/500 (UK), consistent by means of ASTM D 882 (standards). Tests were carried out through a cross-head speed of 12.5 mm min^−1^ until/to a deformation of 20% and then at a speed of 50 mm min^−1^ at break. The gas permeability of the polymer membranes with thickness around 30 mm was measured with an automated Diffusion Permeameter (DP-100-A) manufactured by Porous Materials Inc., USA, which consists of upstream and downstream parts separated by a membrane. Gases measured include N_2_ and CO_2_. The permeation cell was placed in a thermostatically controlled housing for maintaining isothermal measurement conditions. The reproducibility of the measurements was checked from three independent measurements using the same membrane, and it was better than ±5%.

### 2.2 Starting materials

5-bromo-2-methylisoindoline-1, 3 dione, *p*-toluidine and tetrakis(triphenylphosphine) palladium (0) were purchased from Alfa Aesar and used as received. Commercially available N-methyl-2-pyrrolidinone (NMP), m-cresol, N, N-dimethylacetamide (DMAc), N,N-dimethylformamide (DMF), dimethyl sulfoxide (DMSO), tetrahydrofuran (THF) and other reagents were all used as received. TiO_2_ nanoparticles with an average particle size of about 30–50 nm were purchased from Neutrino Co (Tehran, Iran). Nitrogen and Carbon dioxide gases from BOC were used for the permeation study. The cellulose nanofibers (CNFs) used in this study were provided by the Institute of Tropical Forestry and Forest Products (INTROP), Malaysia, and were isolated from the kenaf bast fibers (Hibiscus cannabinus). The details of the CNFs isolation process are reported elsewhere [48]. The selected fungus was a white rot fungus (Trametes versicolor), which was obtained from the National Collection of Biology Laboratory, University of Tehran, Iran. Glycerol, methanol, acetone, acetic anhydride (95%), pyridine, and malt extract agar (MEA) were purchased from the Merck Chemical Co., Germany. All the materials and solvents that were used were obtained from the suppliers without further purification.

### 2.3 Gas transport test

The permeability of oxygen, nitrogen, methane and carbon dioxide was determined using constant pressure/variable volume method at 4 bar pressures and at 25 °C. The gas permeability of membranes was determined using the following equation:

$$P=\frac{\mathrm{ql}}{A(P_{1}-P_{2})}$$

where *P* is permeability expressed in Barrer (1 Barrer = 10^−10^ cm^3^ (STP) cm/cm^2^ s cmHg), *q* is flow rate of the permeate gas passing through the membrane (cm^3^/s), *l* is membrane thickness (cm), *p*_1_ and *p*_2_ are the absolute pressures of feed side and permeate side, respectively (cmHg) and *A* is the effective membrane area (cm^2^).

The ideal selectivity, α_A/B_ (the ratio of pair gas permeabilities) of membranes was calculated from pure gas permeation experiments.

$$\alpha_{A/B}=\frac{P_{A}}{P_{B}}$$

### 2.4 Biodegradation test

In order to study the fungal degradation of the bionanocomposites, a white rot fungus (T. versicolor) was used. The specimens of the pure PI and PI/BNCs (5, 10 and 15%) nanocomposites were prepared with lateral dimensions of 20.0 × 10.0 × 0.4 mm^3^ (length × width × thickness). The samples were dried at 70 °C in an oven overnight and the initial weight of each specimen was recorded. The purified fungus was transferred to the Petri dishes containing MEA. The dishes were then kept in the laboratory incubator at 25 °C until the culture medium was fully covered by the fungus. The specimens were then transferred into the Petri dishes containing the culture medium. To prevent direct contact of the specimens with the culture medium, the specimens were mounted over two 2-mm platforms. The Petri dishes containing the fungus and the specimens were then stored in an incubator at 25 °C and 75% RH. The biodegradation rate of the specimens were evaluated for two months and at regular intervals of 10 days by weight differences before and after the exposure of the specimens to the white rot fungi. The fungal degradation rate was calculated using below equation:

$$\mathrm{DE}\;(\%)=\frac{{\text{W}}_{0}-{\text{W}}_{1}}{{\text{W}}_{0}}\times 100$$

where DE is the biodegradation rate of PI, W_0_ is the initial weight of the original specimen, and W_1_is the dry weight of the residual specimen exposed to the white rot fungi for a certain time.

### 2.5 Monomer synthesis

The diimide compound 1 obtained from double N-arylation reactions of *p*-toluidine with 5-bromo-2-methylisoindoline-1, 3-dione was carried out in the presence of palladium (II) acetate, *rac*-2,2′-bis(diphenylphosphino) -1,1′-binaphthyl (*rac*-BINAP), and cesium carbonate in toluene. The resulting diimide compound (1) was then hydrolyzed with aqueous potassium hydroxide, giving the corresponding tetracarboxylic acid, which in turn was converted to the new dianhydride monomer 2 by the chemical cyclodehydration with acetic anhydride (Scheme 1). Elemental analysis, FT-IR, NMR and ^13^C NMR spectroscopic techniques were used to identify structures of the dianhydride monomer. The carbonyl groups of diimide compound exhibit two characteristic bands at around 1721 and 1657 cm^−1^ could be attributed to imide C=O asymmetric and symmetric stretching, respectively. After hydrolyzed and cyclodehydrated to dianhydride monomer, the carbonyl groups shifted to around 1825 and 1715 cm^−1^. Fig. 1 illustrates the NMR and ^13^C NMR spectra of the dianhydride monomer 2 and these spectra agree well with the proposed molecular structure. Thus, the results of all the spectroscopic and elemental analyses suggest the successful preparation of the target dianhydride monomer 2.

**Scheme 1:** Synthesis of monomer dianhydride and Synthesis of PI with a trifluoromethyl pendent group.

**Fig. 1:** ^1^H NMR (500 MHz) spectrum of dianhydride (2) in DMSO-*d*_6_ at R.T and ^13^C NMR (125 MHz) spectrum of dianhydride (2) in DMSO-*d*_6_ at R.T.

**FT-IR (compound 1) (KBr, cm^−1^):** 3156 (w), 3063 (w), 2955 (s), 2913 (w), 1721 (s), 1657 (s), 1525 (s) 1424 (m), 1331 (m), 1121 (w), 855 (m), 658 (w).

**FT-IR** (**compound 2) (KBr, cm^−1^):** 3158 (w), 3075 (w), 2951 (w), 2901 (w), 1825 (s), 1715 (s), 1622 (s) 1424 (m), 1344 (m), 1169 (w), 825 (m), 715 (w).

**^1^H NMR (compound 2) (500 MHz, DMSO-*d_6_*, ppm):** 2.31 (s, 3H, C-H), 7.13–7.15 (d, 2H, Ar-H, *J* = 4.0), 7.25–7.27 (d, 2H, Ar-H, *J* = 4.0), 7.42–7.44 (d, 2H, Ar-H, *J* = 4.0), 7.56 (s, 2H, Ar-H), 7.66–7.68 (d, 2H, Ar-H, *J* = 4.0).

**^13^C NMR (compound 2) (125 MHz, DMSO-*d_6_*),** δ (ppm): 28.53 (CH_3_), 118.42 (Ar), 124.62 (Ar), 128.43 (Ar), 131.21 (Ar), 133.32 (Ar), 134.31 (Ar), 138.12 (Ar), 140.98 (Ar), 141.25 (Ar), 168.24 (C=O).

**Elemental analysis (compound 2): calcd. For C_23_H_13_NO_6_** (399.07 g mol^−1^): C, 69.17%; H, 3.28%; N, 3.51%. Found: C, 68.82%; H, 3.22%; N, 3.78%.

### 2.6 Polymer synthesis

PI was prepared by the one/pot, high/temperature solution polymerization of dianhydride monomer with aromatic diamine in m-cresol at 200 °C in the presence of isoquinoline as the catalyst (Scheme 1). Polymerization reaction proceeded homogenously and led to the formation of highly viscous polymer solutions that can be precipitated into tough fiber-like forms when slowly trickling into methanol. The resulting PI exhibited inherent viscosities of 1.67 dL/g in N-methyl-2-pyrrolidinone (NMP) and can afford transparent/self/standing films via solution casting, indicating this is high molecular weight polymer. Moreover, the number average molecular weight (M_n_), weight average molar weight (M_w_) and polydispersity index (PDI) of the synthesized polymer was further supported by GPC measurements. The structure of these PI was also confirmed with IR and NMR spectroscopic techniques, and the spectra agree well with the proposed molecular structures. The IR spectra of PI exhibit characteristic imide absorption bands at around 1775 (imide asymmetrical C=O), 1727 (imide symmetrical C=O), 1355 (C—N), and 755 cm^−1^ (imide ring deformation) (Fig.2(a)). A typical ^1^H NMR spectrum of PI shown in Fig.2(b) reveals that all the peaks could be readily assigned to the hydrogen atoms of the recurring unit.

**Fig. 2:** (a) FT-IR spectrum of the PI and (b) ^1^H NMR (500 MHz) spectrum of PI in DMSO-*d*_6_ at RT.

PI was also characterized by elemental analysis techniques, and the results are in good agreement with the calculated ones for the proposed structures. These results in sum confirmed the successful formation of the new PI.

**FTIR (KBr, cm^−1^)**: 3450 (m, br), 3125 (w), 2920 (w), 1775 (m), 1727 (s), 1650 (m), 1550 (s), 1475 (s), 1387 (s), 1355 (s), 1319 (s), 975 (s), 952 (m), 850 (m), 735 (m), 725 (m), 660 (m), 560 (m).

**^1^H NMR (400 MHz, DMSO-*d_6_*, ppm):** 2.35 (s, 3H, C-H), 7.24–7.25 (d, 2H, CH, *J* = 3.6 Hz), 7.34–7.36 (d, 2H, Ar-H, *J* = 6.4 Hz), 7.52–7.55 (d, 2H, Ar-H, *J* = 8.4), 7.57–7.59 (d, 2H, Ar-H, *J* = 4.0), 7.67 (s, 2H, Ar-H), 7.77–7.79 (d, 2H, Ar-H, *J* = 6.2), 7.89–7.91 (d, 2H, Ar-H, *J* = 5.4).

**GPC measurements of resulting PI: M_n_** 84 123, M_w_: 185 194, PDI: 2.20.

**Elemental analysis calculated for C_38_H_22_F_6_N_3_O_4_** (698.15 g mol^−1^): C, 65.33%; N, 6.01%; H, 3.17%, Found: C, 64.83%; H, 3.16%; N, 6.21%.

### 2.7 Surface functionalization of TiO_2_ nanoparticles with nanofiber cellulose

Nanofiber cellulose was modified TiO_2_ nanoparticle by ultrasonic irradiation. Typical steps were given as follows: nanoTiO_2_ was dried at 120 °C in an oven for 24 h to remove the adsorbed water. 0.10 g of dried nanoTiO_2_ in DMF solution by a sonication treatment for 20 min (through an ultrasonic instrument MISONIX, 100 W), then 0.05 g of nanofiber cellulose was added to this mixture and sonicated for 45 min. The mixture was filtered and dried at 75 °C for more than 24 h.

### 2.8 Preparation of the PI/BNCs

The PI/BNCs were synthesized via mixing the 0.1 g PI with different amounts of modified TiO_2_ (cellulose/TiO_2_) (5, 10, and 15 wt%) in 25 mL of DMF followed by irradiation with high-intensity ultrasonic wave for 8 h. After irradiation, the solvent was removed and the obtained solid was dried in vacuum at 130 °C for 4 h. (Scheme 2).

**Scheme 2:** Reaction of TiO_2_ nanoparticles with cellulose and Preparation of PI/BNCS.

## 3 Results and discussion

### 3.1 FT-IR studies of the BNCs (cellulose/TiO_2_) films

FT-IR studies were carried out to confirm the identification and bond structure of associated functional groups of as-synthesized TiO_2_ impregnated cellulose using optimized parameters. The infrared absorption spectra of cellulose, TiO_2_ NPs and cellulose/TiO_2_ nanocomposites were observed in the 4000–400 cm^−1^ wave-number range (Fig. 3). Comparison of citrus cellulose and TiO_2_ NPs with that of cellulose/TiO_2_ composite demonstrates an appropriate coincidence. The intermolecular hydrogen bonds in cellulose may be weaker than those in the cellulose/TiO_2_ and the low crystallinity and intermolecular hydrogen bonds in cellulose make it more reactive component when participating in a chemical reaction.

**Fig. 3:** (a) FT-IR spectra of pure TiO_2_ nanoparticle, (b) pure cellulose and (c) modified TiO_2_ nanoparticle.

The FT-IR spectrum of TiO_2_ (Fig.3a) show main absorption bands at 3450, 1580, and 1375 cm^−1^, which correspond to the O—H mode, and peak at 437 cm^−1^is the characteristic absorption of Ti—O bond. In the cellulose spectrum (Fig.3b), the stretching and bending modes of the —OH group were viewed at 3435 and 1575 cm^−1^, respectively. The peak at 1030 cm^−1^ originates from the C—O stretching of cellulose. Such results and appeared new bands at 2885 cm^−1^in the FT-IR spectrum of modified TiO_2_ nanoparticles indicate that the cellulose have been successfully grafted onto the surface of TiO_2_ nanoparticles.

### 3.2 XRD analysis of the BNCs films

XRD analyses were conducted to investigate the crystallinic properties of cellulose, the synthesis of cellulose/TiO_2_ nanocomposites and the micro-structural changes in the cellulose sheets caused by the TiO_2_ nanoparticles. Fig. 4 shows the XRD patterns of the pure cellulose (a), pure TiO_2_ (b) and cellulose/TiO_2_ (c). The characteristic peaks of cellulose appeared at 2θ values of 23.1° and 34.9° corresponds to the structure of planes particles [50], [51]. Neither a new peak nor a peak shift compared with the pure cellulose indicates that the cellulose/TiO_2_ nanocomposite films consist of two phase structures that may be polymer and nanoparticles. These observations show that the addition of the cellulose/TiO_2_ causes an overall increase in crystallinity of pure PI that can be effective on the final proprieties of biocomposites films.

**Fig. 4:** (a) XRD spectra of pure cellulose, (b) pure TiO_2_ nanoparticle and (c) modified TiO_2_ nanoparticle.

### 3.3 SEM and TEM analysis of the BNCs films

The formation of TiO_2_ NPs on the surface of cellulose can be observed as scattered molecules on the surface of cellulose with <100 nm size (Fig.5a and b). Fig. 5 presents a microscopic image shown at different magnifications. The research on nanoscale materials demonstrate various sizes of particles produced. The nanocrystalline microstructure of TiO_2_ has a skeletal form subsequent to the procedure of coagulation (Fig. 2). Natural cellulose has non-woven network with large number of pores. According to the SEM photographs of cellulose/TiO_2_ reveal that the TiO_2_ nanoparticles were dispersed in the cellulose and the average particle size of the nanoparticles was in the range of 35–38 nm (Fig.5a and b). TEM has confirmed to be a powerful tool for studying the dispersion of nanofillers embedded within a cellulose matrix. The TEM micrograph of the cellulose/TiO_2_ shows that nanoparticles were dispersed in the cellulose matrix and some aggregation maybe observed in the TEM images (Fig.5c and d).

**Fig. 5:** SEM and TEM analysis of the BNCs (cellulose/TiO_2_) films.

### 3.4 FT-IR analysis of PI/BNCs

The incorporation BNCs in PI caused the slight changes in the intensities of absorption bands to 1725 and 1675 cm^−1^ as well as the formation of new absorption bands in the range of 400–700 cm^−1^. Peak around 400–700 cm^−1^ is attributed to the Ti—O stretching of TiO_2_. This corroborated the presence of TiO_2_ nanoparticles present in the PI matrix. This indicates that there is no chemical linkage between PI and BNCs. Therefore, the comparatively weak interaction is thought to be a hydrogen bond, and also short-ranged steric and electrical interaction among active sites of cellulose/TiO_2_ and various functional groups of PI. FT-IR spectrums of PI and BNCs polymers with different amounts of cellulose/TiO_2_ (5, 10, and 15 wt%) show the intensity of TiO_2_ stretching band raise with an increase of cellulose/TiO_2_ content in PAI.

### 3.5 X-ray diffraction of PI/BNCs

Fig. 6 displays the X-ray diffraction (XRD) patterns of BNCs (cellulose/TiO_2_) (a), pure PI (b) and PI/BNCs (10%) (c). The XRD pattern of PI/BNC shows characteristic peaks of PI and cellulose/TiO_2_ indicating that the crystallinity of TiO_2_ nanoparticles was not changed during the preparation process. The average particle size of nanoparticles was estimated based on Scherrer correlation of particle diameter (D) D = K λ/β cos θ where K is the Scherrer constant, λ the X-ray wavelength, β the peak width at half-maximum, and θ is the Bragg diffraction angle. The average crystallite size of the TiO_2_ calculated from the width of the diffraction peak according to the Scherrer equation is approximately less 45 nm. This is in agreement with the size of used TiO_2_ nanoparticles. Pure PI (Fig.6a) was totally amorphous in nature, which did not show any sharp diffraction peaks.

**Fig. 6:** (a) XRD spectra of cellulose/TiO_2_, (b) pure PI and (c) PI/BNCs (10%).

### 3.6 Thermal and mechanical properties of PI/BNCs

The thermal properties of the PI/BNCs were evaluated by means of TGA in a nitrogen atmosphere at a heating rate of 10 °C/min. Table 1 shows the data for the thermal degradation of the PI and PI/BNCs including the temperature at which 5% (T_5_), 10% degradation occurs (T_10_), Limiting oxygen index (LOI) and char yield at 800 °C. LOI values were calculated based on Van Krevelen and Hoftyzer equation [49]. LOI = 17.5 + 0.4 CR where CR = char yield. As shown in Fig.7b, the initial decomposition temperatures of the pure PI and PI/BNCs are about 375 °C. The char yield values of PI/BNCs have higher thermal stability than that of pure PI at 800 °C. Increasing in the thermal stability in PI/BNCs is attributed to the high heat resistance exerted by the TiO_2_, because the TiO_2_ nanoparticles have high thermal stability so coupling of TiO_2_ nanoparticles can improve the thermal stability of the PI/BNCs.

**Table 1:** Thermal characterizations of pure PI and PI/BNCs film.

Polymer	T_5_^a^ (°C)	T_10_^a^ (°C)	Char yield (%)^b^	LOI^c^
PI	355	375	71	45.9
PI/BNC (5%)	385	390	76	47.9
PI/BNC (10%)	395	395	76.5	48.1
PI/BNC (15%)	402	408	77.8	48.62

a Temperature at which 5 and 10% weight loss was recorded by TGA at a heating rate of 10 °C min^−1^ in a nitrogen atmosphere.

b Percentage weight of material left undecomposed after TGA analysis at maximum temperature 800 °C in a nitrogen atmosphere.

c Limiting oxygen index (LOI) evaluating at char yield at 800 °C.

**Fig. 7:** (a) Tensile stress–strain curves of the pure PI and PI/BNCs hybrid films with different amounts of cellulose/TiO_2_ (b) TGA thermograms of PI and PI/BNCs with different cellulose/TiO_2_ content.

The average values and standard deviations of the neat PI and PI/BNCs tensile properties are summarized in Table 2. The tensile properties showed that an increased modulus and strength of both PI/BNCs with 15 wt% BNCs (cellulose/TiO_2_) compared to the pure PI. The effect of adding BNCs on PI matrix is related with the interactions of molecules in the hybrid films. Tensile properties of the PI/BNCs hybrids films were studied by typical stress–strain curves. Specific values of the ultimate properties and the modulus of these samples are shown in Fig.7a and the results are listed in Table 2. In comparison the pure PI with different amount of BNCs has higher ultimate strength; higher initial Young's modulus, but lower ultimate elongation. The ultimate properties of the BNCs are dependent on different parameters, such as the extent of bonding between the polymer matrix as continuous phase and BNCs as discontinuous phase, the surface area of the TiO_2_, and the arrangements between the BNCs. The abovementioned results showed that the interactions between the PI matrix and BNCs are very important in the preparation of hybrid materials.

**Table 2:** Mechanical properties for pure PI with various BNCs.

Material	Modulus^a^ (MPa)	Ultimate strength^b^ (MPa)	Ultimate elongation^c^ (%)
PI	3312.54	230.44	11.92
PI/BNC (5%)	3544.32	238.56	10.22
PI/BNC (10%)	3675.98	247.87	9.32
PI/BNC (15%)	3698.43	257.12	8.26

a Initial slope of the stress–strain curve.

b Stress at break.

c Elongation at break.

### 3.7 Electron microscope characterization of PI/BNCs

Fig.8a and b shows the FE-SEM micrographs of PI/BNC (10 wt%). The average particle size of the nanoparticles was in the range of 45–55 nm. The FE-SEM images of PI/BNC (15 wt%) reveal that the cellulose/TiO_2_ BNCs were homogeneously dispersed in the polymer matrix. Due to treating TiO_2_ filler with modifying agents such as cellulose and ultrasound irradiation that effect on the distribution and particle size of the nanoparticles the compatibility of TiO_2_ filler with PI matrix are able to be improved.

**Fig. 8:** (a) and (b) FE-SEM micrograph PI/BNC 10%, (c) and (d) TEM micrographs of PI/BNC 10%.

TEM has confirmed to be a powerful tool for studying the dispersion of nanocomposits embedded within a polymer matrix. The TEM micrograph of the PI/BNC (10 wt%) in Fig.8c and d shows that BNCs were homogeneously dispersed in polymer matrix. The modified BNCs (cellulose/TiO_2_) might be dispersed absolutely and will combine with PI via the H-bonding of NH_2_ coupling agent with —NH, C=O, groups in PI. In addition —OH groups on the surface of TiO_2_ nanoparticle can bond to the amide group (C=O) of PI through interchange hydrogen bonding. The average size of the nanoscale TiO_2_ particles is about 45 nm. The obtained results show that the surface modification plays a main role in dispersion of nanoparticles.

### 3.8 Gas permeation results of PI/BNCs

The permeation of N_2_, CH_4_, H_2_ and CO_2_ in pure PI and PI/BNCs membranes was investigated at ambient temperature and pressure of 4 × 10^5^ Pa. The results of gas permeation properties of PI/BNCs membranes are illustrated in Table 3 and Fig. 9, Fig. 10. As shown in this table, the permeability of carbon dioxide increases from 75.43 × 10^−16^ to 114.62 × 10^−16^ mol m/(m^2^ s Pa) and the permeability of hydrogen and nitrogen increase from 89.23 × 10^−16^ and 2.44 × 10^−16^ to 126.65 × 10^−16^ and 3.73 × 10^−16^ mol m/(m^2^ s Pa), respectively. By comparison of our results with targeted papers [50], [51], we can see that the membranes prepared achieved convenient results. Gas solubility, gas molecular size, void volume in the polymer and also the mobility of the polymer chains are the main properties of polymeric membranes that affect the permeability of gases through the polymer. In the glassy polymers such as PI, due to their rigid structure and the vacancy of chain mobility, the permeation of the gases in the polymer is defined by the diffusivity ability of the gases in the polymer [52].

**Table 3:** Gas permeabilities of PI and PI/BNCs membranes as a function of TiO_2_ at ambient temperature and 4 bar.

Membrane name	Permeability (×10^−16^ mol/m^2^ s Pa)			
	H_2_	CO_2_	N_2_	CH_4_
Pour PI	89.52	75.43	2.35	1.62
PI/BNC (5%)	116.87	97.64	3.22	2.73
PI/BNC (10%)	121.43	108.21	3.43	3.12
PI/BNC (15%)	126.65	114.62	3.73	3.48

1 barrer = 3.34 × 10^−16^ (mol m/m^2^ s Pa).

**Fig. 9:** The comparison of gas permeability of N_2_ and CH_4_ for PI/BNCs membranes.

**Fig. 10:** The comparison of gas permeability of H_2_ and CO_2_ for PI/BNCs membranes.

Generally, incorporation of BNCs (cellulose/TiO_2_) in a glassy polymer matrix can disrupt its chain packing, which increases the free volume in the polymer phase. In addition, voids at the polymer particle interface or between particles in particle aggregates result in an increase in total free volume. Increased total free volume leads to increases in diffusion and solubility coefficients and thus causes gas permeability to be greater in BNCs than in pure polymer. Fractional free volumes (FFVs) for all the PI/BNCs membranes with respect to four different gases were estimated using group contribution method developed by Park and Paul [53]. The order of fractional free volume for the PI/BNCs membranes for all the gases was PI/BNC (15%) > PI/BNC (10%) > PI/BNC (5%) > Pure PI (Table 4). Incorporation of BNCs in the polymer matrix is known that PI/BNC (15%) has higher fractional free volume in the series. The order of gas permeability coefficients of four PI/BNCs membranes for all the gases was PI/BNC (15%) > PI/BNC (10%) > PI/BNC (5%) > Pure PI. The dependence of permeability coefficients with FFV of the PIs for the four gases (CO_2_, H_2_, N_2_ and CH_4_) is represented in Table 4.

**Table 4:** Fractional free volumes and observed density of the PI/BNCs.

Membrane name	Free volumes			
	FFV^a^_H2_	FFV^a^_CO2_	FFV^a^_N2_	FFV^a^_CH4_
Pour PI	0.20	0.16	0.19	0.18
PI/BNC (5%)	0.24	0.22	0.21	0.21
PI/BNC (10%)	0.27	0.23	0.23	0.26
PI/BNC (15%)	0.28	0.23	0.28	0.28

a FFV = [V − (V_o_)_n_]/V, where V is the volume per mole of the repeat unit of the polymer at 30 °C, (V_o_)_n_ = ∑γ_nk_(V_w_)_k_, γ_nk_ is set of empirical factors depending upon gas ‘n’ and group ‘k’. (V_w_)_k_ represents van der Waals volumes for group ‘k’ [53].

In PI/BNCs membranes, nonporous TiO_2_ nanoparticles substitute some portions of the dense and porous structure of the polymer matrix. It can be also observed from the FE-SEM and TEM that voids have been formed at the PI/BNCs interface. Table 3 presents the gas permeability of pure PI and PI/BNCs membranes. As can be seen in Table 3, by increasing TiO_2_ loading, gas permeability increases. This trend is similar to those reported for a variety of non-porous nanoparticle fillers dispersed in glassy polymers. The separation performance of membranes was calculated for selected gas pairs. The ideal gas selectivities of TiO_2_-filled membranes are listed in Table 4. These data indicate that the selectivity of pairs of gases decreases with TiO_2_ content. Results suggested that void volume was formed at the interface between polymer and TiO_2_ nanoparticles due to the agglomeration of the nanoparticles observed in polymer matrix by FE-SEM and TEM.

### 3.9 Biodegradability of composites

The biodegradability of the pure PI and PI/BNCs (5, 10 and 15%) nanocomposites was investigated undertaking white rot fungi (T. versicolor) at regular time intervals by measuring the weight loss. Table 5 shows the degradation process and the weight loss with respect to the elapsed time. By increasing the decomposition time, the compactness of the films would be reduced. Fig. 11 shows weight remaining of biodegradability test for pure PI and PI/BNCs (5, 10 and 15%) nanocomposites according to days. Accordingly, it was observed that the degradation occurred in a faster rate in the presence of cellulose/TiO_2_ in the PI matrix. Consequently, the BNCs could be easily degraded in natural condition (see Table 6).

**Table 5:** The ideal selectivity of pure PI and PI/BNCs membranes with different TiO_2_ loadings.

Membrane name	Ideal selectivity		
	H_2_/N_2_	H_2_/CO_2_	CO_2_/CH_4_
Pour PI	38.10	1.18	46.56
PI/BNC (5%)	36.22	1.19	35.76
PI/BNC (10%)	35.40	1.12	34.68
PI/BNC (15%)	33.95	1.10	32.93

**Fig. 11:** Weight loss of biodegradability test for pure PI and PI/BNCs (5, 10 and 15%) nanocomposites according to days.

**Table 6:** Biodegradation for the pure PI and PI/BNCs films.

Films	Weight loss (g)			
	10 day	20 day	45 day	60 day
Pure PI	0.19	0.10	0.08	0.04
PI/BNC (5%)	0.32	0.12	0.09	0.05
PI/BNC (10%)	0.43	0.10	0.07	0.05
PI/BNC (15%)	0.55	0.11	0.06	0.07

## 4 Conclusions

PI/BNCs have been prepared by irradiation with high-intensity ultrasonic wave. FT-IR spectral measurements allow us to conclude that polymer bionanocomposite has formed and also there is intermolecular interaction between the PI and cellulose/TiO_2_. The thermal analysis depicts the percentage of the inorganic material in an organic matrix. The thermal stability of the PI/BNCs has increased compared to that of pure PI. TEM and FE-SEM images confirmed the dispersion of cellulose/TiO_2_ in the polymer matrix. The gas separation properties of PI membrane with three cellulose/TiO_2_ concentrations (5, 10 and 15 wt%) are tested for gas permeation. The permeability and selectivity of the PI/BNCs membranes as a function of the titania weight percentage were study and the results indicated that the permeabilities of CO_2_, H_2_, CH_4_ and N_2_ increase with increasing TiO_2_ concentration.
